The article "The COVID-19 fear, anxiety, and resilience among emergency nurses" was retracted in 2023. Reasons: signs of a paper mill; concerns about the authorship.

# The COVID-19 fear, anxiety, and resilience among emergency nurses

**DOI:** 10.3389/fpsyg.2022.999111

**Published:** 2022-09-02

**Authors:** Negar Karimi Khordeh, Fazel Dehvan, Sahar Dalvand, Selman Repišti, Reza Ghanei Gheshlagh

**Affiliations:** ^1^Student Research Committee, Kurdistan University of Medical Sciences, Sanandaj, Iran; ^2^Clinical Care Research Center, Research Institute for Health Development, Kurdistan University of Medical Sciences, Sanandaj, Iran; ^3^Department of Epidemiology and Biostatistics, School of Public Health, Tehran University of Medical Sciences, Tehran, Iran; ^4^Psychiatric Clinic, Clinical Center of Montenegro, Podgorica, Montenegro; ^5^Social Determinants of Health Research Center, Research Institute for Health Development, Kurdistan University of Medical Sciences, Sanandaj, Iran

**Keywords:** emergency nurses, COVID-19 fear, COVID-19 anxiety, resilience, COVID-19

## Abstract

**Background:**

Besides physical complications, COVID-19 is associated with psychological issues such as fear and anxiety. High resilience in nurses enables them to adopt positive coping mechanisms and successfully operate in the stressful environment of COVID-19 wards. The present study aimed to evaluate the correlation between COVID-19 fear and anxiety with resilience in the emergency nurses of the hospital affiliated with Kurdistan University of Medical Sciences (west of Iran) in 2021.

**Materials and methods:**

This cross-sectional study was conducted on 295 emergency nurses of selected hospitals in Kurdistan province, Iran, in 2021. Data were collected using a demographic questionnaire, Fear of COVID-19 Scale (FCV-19S), Corona Disease Anxiety Scale (CDAS), and Connor-Davidson Resilience Scale (CD-RISC). Data analysis was performed in R software version 3.6.3.

**Results:**

The mean scores of resilience, COVID-19 fear, and COVID-19 anxiety were 55.07 ± 19.82 (ranging from 0 to 100), 20 ± 7.37 (ranging from 7 to 35) and 36.48 ± 13.21 (ranging from 18 to 54) respectively. There was a negative and significant correlation between resilience with COVID-19 fear (*r* = −0.449, *p* = 0.001), COVID-19 anxiety (*r* = 0.458, *p* = 0.001). A significant correlation was observed between COVID-19 fear and anxiety, which indicated that if the other demographic variables remained unchanged, a one-unit increase in COVID-19 fear and anxiety decreased the mean resilience score by −0.66 (*P* = 0.008) and −0.34 (*P* = 0.015), respectively.

**Conclusion:**

COVID-19 fear and anxiety were significantly correlated. Therefore, providing training courses for promoting resilience could reduce the fear and anxiety of nurses during the COVID-19 pandemic.

## Introduction

The coronavirus disease 2019 (COVID-19) pandemic was first reported in Hubei Province of China in December 2019 and has currently affected approximately six million, leading to a high mortality rate (Luo et al., 2021). On March 11, 2020, the World Health Organization (WHO) declared the coronavirus disease a pandemic, and the world entered a new phase of battling the disease (Pakzad and Owlia, 2020). The current pandemic has imposed unprecedented pressure on the healthcare system, causing numerous challenges for healthcare providers (especially nurses), adversely affecting their professional performance and psychological health (Imani Jaajarmi, 2020; Labrague and De los Santos, 2020). The nature of the disease is associated with severe stressful reactions, such as fatigue, depression, fear, and anxiety in the general population and even healthcare providers, particularly nurses (Asadi et al., 2020). The nurses’ workload has increased tremendously with the emergence of COVID-19 and the frequent referral of patients to health centers (Moradzadeh and Joyami, 2020).

Emergency department nurses are the frontline healthcare workers in the COVID-19 pandemic (Abadi et al., 2020). Nurses have experienced the highest anxiety levels among various healthcare professionals, estimated at 15-92% (Alwani et al., 2020). COVID-19 fear and anxiety in emergency nurses are caused by several factors, including direct contact with COVID-19 patients (Pappa et al., 2020), fear of disease transmission to oneself and one’s family members, handling new and changing treatment protocols, shortage of personal protective equipment (Walton et al., 2020), heavy workload, extensive media coverage, lack of specific medications, and lack of adequate support (Lai et al., 2020). Although low levels of anxiety could benefit motivation and excitement, persistent exposure to unmanaged anxiety adversely affects physio-psychological health and work performance while also causing job dissatisfaction, frequent absenteeism, and nurse turnover (Labrague, 2018; Lee, 2020).

Resilience could influence the stress and anxiety levels of those exposed to the coronavirus (Vakili et al., 2020). Resilience refers to a person’s capacity to “bounce back” or recover quickly from a stressful event (Hart et al., 2014), which could help nurses confront stressors effectively and endure the burden caused by these stressors. Resilience is a major contributing factor to adaptation to change and the ability to resist the issues and complications associated with COVID-19 (Pourafzal et al., 2013).

Nurses must attempt to develop resilience to endure professional hardships, overcome negative experiences, and turn such experiences into positive ones. Otherwise, work conditions will become intolerable to nurses, and they might suffer psychological and environmental issues, which make working in the environment problematic (Gerami Nejad et al., 2018). While numerous harmful occupational factors could affect nurses under normal circumstances, the emergence of COVID-19 and its rapid spread may be associated with fear and anxiety in these healthcare professionals.

The present study aimed to evaluate the correlation between COVID-19 fear and anxiety and resilience in the emergency nurses of the hospitals affiliated with the Kurdistan University of Medical Sciences (west of Iran) in 2021.

## Materials and methods

### Design and setting

This cross-sectional study was conducted with the nurses employed in the emergency department of the hospitals affiliated with the Kurdistan University of Medical Sciences (west of Iran). The participants were selected *via* convenience sampling. Convenience sampling is a non-random sampling in which researchers collect data from a pool of available respondents. Convenience sampling is the most common method because it is speedy, uncomplicated, and cost-effective. The sampling process lasted from October 9, 2021, to November 8, 2021, which coincided with the third wave of COVID-19 in Iran. Two inclusion criteria had to be met, being employed in the emergency ward during the COVID-19 pandemic and having more than 1 year of clinical experience. Incomplete questionnaires were eliminated. According to Kendall’s principle, at least 10 participants are needed for each variable (Lewis, 2009). Considering that the number of variables in this study was 15, we considered 20 samples for each variable, so our sample size was 295 people.

### Measurement

Data were collected using a demographic questionnaire, the Fear of COVID-19 Scale (FCV-19S), the Corona Disease Anxiety Scale (CDAS), and the Connor-Davidson Resilience Scale (CD-RISC).

### Questionnaire on demographic and some COVID-19 related variables

This questionnaire included data on age, gender, marital status, work experience, type of employment, education level, previous training on COVID-19, history of COVID-19 vaccination, and history of COVID-19 infection.

#### Fear of COVID-19 scale (FCV-19S)

The FCV-19S has been developed by Ahorsu et al. (2020) with seven items, which are scored based on a five-point Likert scale (Completely disagree = 1, Completely agree = 5). The final score of the scale is calculated within the range of 7–35, and higher scores indicate more fear (Ahorsu et al., 2020). The original version of the FCV-19S is available in English and Persian. After obtaining permission from the original designer, we used the Persian version of this tool to assess the fear of COVID-19. In our study, the reliability of the scale was estimated at 0.92.

#### Corona disease anxiety scale (CDAS)

Alipour et al. (2020) prepared this scale in the Farsi language, which has 18 items with four-point Likert responses (never = 0, always = 4) (Alipour et al., 2020). Higher scores on the CDAS indicate much anxiety. In the initial study, the reliability of the scale was confirmed with Cronbach’s alpha coefficient of 0.919 (Alipour et al., 2020). In the present study, Cronbach’s alpha coefficient of this tool was 0.954. To use this tool, we got permission from the original designer.

#### Connor-Davidson resilience scale (CD-RISC)

Connor and Davidson have developed this tool with 25 items, which are scored on a five-point Likert scale (Never = 0, Always = 4). The final score of the scale is calculated within the range of 0–100, and higher scores indicate more resilience (Connor and Davidson, 2003). In another classification, scores below 71 show poor resilience, scores 71–91 indicate moderate resilience, and scores above 91 show high resilience (Connor and Davidson, 2003; Davidson, 2018). In the present study, the Cronbach’s alpha coefficient of the CD-RISC was 0.956.

### Statistical analysis

Data analysis was performed in R software version 3.6.3. Quantitative variables were described and reported with mean and standard deviation, and qualitative variables with frequency and percentage. In addition, a sex- and age-adjusted multiple linear regression model was used to evaluate the correlation between resilience and the study variables. In all the statistical analyses, the significance level was set at 0.05.

### Ethics approval and consent to participate

The Ethics Committee of the Kurdistan University of Medical Sciences has approved this study (IR.MUK.REC.1400.174). All procedures were performed in this study following the 2013 Declaration of Helsinki. Consent was obtained from all participants.

## Results

In total, 295 nurses (140 males and 155 females) with a mean age of 30.37 ± 5.46 years and a mean work experience of 6.48 ± 5.28 years were enrolled in the study. The majority of the participants were female (52.5%) and married (58.6%), had a bachelor’s degree (92.2%) and history of COVID-19 infection (70.2%), and were vaccinated (89.8%). Table 1 provides more details in this regard.

**TABLE 1:** Distribution of the participants according to demographic and some COVID-19 related data.

Variable	Frequency	Percentage
**Gender**		
Male	140	47.5
Female	155	52.5
**Marital status**		
Married	173	58.6
Single	122	41.4
**Type of employment**		
Permanent	50	16.9
Conditional	79	26.8
Contract	44	14.9
Mandatory	122	41.4
**Training course**		
Yes	94	31.9
No	201	68.1
**Vaccine**		
Yes	265	89.8
No	30	10.2
**History of Covid-19**		
Yes	207	70.2
No	88	29.8

According to the findings, the mean scores of resilience, COVID-19 fear, and COVID-19 anxiety were 55.07 ± 19.82 (ranged from 0 to 100), 20 ± 7.37 (ranged from 7 to 35), and 36.48 ± 13.21 (ranged from 18 to 54), respectively. Based on the scores obtained and obtainable, it can be said that the nurses’ resilience, fear, and anxiety were low to moderate. The Pearson correlation test results showed a negative and significant correlation between resilience with COVID-19 fear (*r* = −0.449, *p* = 0.001) and COVID-19 anxiety (*r* = 0.458, *p* = 0.001). According to multiple linear regression analysis results, none of the clinical demographic and COVID-19-related variables were correlated with the emergency nurses’ resilience. However, COVID-19 fear and anxiety were correlated with resilience. This finding implied that if the other demographic variables remained unchanged, a one-unit increase in the score of COVID-19 fear decreased the mean score of resilience by −0.66 (*p* = 0.008). Also, with an increase of one unit in the COVID-19 anxiety score, the mean resilience score decreases to −0.34 (*p* = 0.015) (Table 2).

**TABLE 2:** Age and sex adjusted multiple linear regression model.

Variable	Coefficient	Std. Error	95% Confidence Interval		*P*-value
			Lower	Upper	
**Marital status (Married)**					
Single	3.73	2.37	−0.94	8.41	0.117
**Type of employment (Mandatory)**					
Permanent	4.93	4.72	−4.37	14.22	0.297
Conditional	−2.80	2.93	−8.57	2.98	0.341
Contract	−0.64	3.46	−7.46	6.18	0.854
**Training course (No)**					
Yes	−4.39	2.36	−9.03	0.26	0.064
**Vaccine status (Vaccinated)**					
Unvaccinated	0.94	3.39	−5.74	7.62	0.782
**History of COVID-19 (No)**					
Yes	−1.04	2.31	−5.59	3.51	0.782
Work experience (Year)	0.08	0.64	−1.19	1.35	0.900
Fear	−0.66	0.24	−1.14	−0.17	0.008
Anxiety	−0.34	0.14	−0.61	−0.07	0.015

## Discussion

The present study aimed to evaluate the correlation between COVID-19 fear and anxiety with resilience in the emergency nurses of the hospitals affiliated with the Kurdistan University of Medical Sciences. According to the results, resilience was significantly correlated with COVID-19 fear and anxiety. This finding implied that if the other underlying and demographic variables remained unchanged, a one-unit increase in the fear and anxiety scores decreased the resilience score by −0.63 and −0.35, respectively. The results of the present study are consistent with the previous findings in this regard (Amirfakhraei et al., 2020; Brooks et al., 2020; Eyni et al., 2020; Wang et al., 2020). Other studies have also identified the protective role of resilience in disaster events (Labrague, 2018) and disease outbreaks (Duncan, 2020), as this quality could help nurses cope with and manage stressful situations. According to the study by Yıldırım and Güler (2021), resilience is an intermediary factor in the correlation between COVID-19 fear and anxiety (Yıldırım and Güler, 2021). In another research, Huffman et al. (2021) reported that resilience is a protective factor against stress and other negative psychological factors resulting from the COVID-19 pandemic in healthcare workers (Huffman et al., 2021).

The study by Kim et al. (2021), which was conducted during the COVID-19 pandemic, also indicated that resilience is a strong predictor of mental health problems in nurses, and the risk of psychological disorders was 2–6 times lower in nurses with higher levels of resilience (Kim et al., 2021). Furthermore, Zhang et al. (2020) reported that resilience was a protective factor for anxiety and stress and decreased depression (Zhang et al., 2020). Several studies performed in the COVID-19 pandemic on healthcare workers have also shown a negative correlation between depression, burnout, and job stress (Jose et al., 2020; Di Giuseppe et al., 2021; Yörük and Güler, 2021). Researchers believe that increasing resilience could protect individuals against the stressors and anxieties that lead to psychological problems in the long run (Rasic et al., 2011; Beheshti and Zarqam Hajabi, 2018).

In the present study, the emergency nurses had a low level of resilience, which is consistent with the results obtained by Roberts et al. (2021). On the other hand, the findings of Luceño-Moreno et al. (2020) in Spain during the COVID-19 pandemic indicated moderate resilience in healthcare personnel (Luceño-Moreno et al., 2020). Previous findings in the COVID-19 pandemic have also confirmed the moderate resilience of nurses (Afshari et al., 2021; Ou et al., 2021). According to Sinu Jose et al. (2020), frontline COVID-19 nurses in India had moderate-to-high resilience (Jose et al., 2020). Resilience is a complex and dynamic process affected by personal characteristics, environmental/social factors, and profession (Cooper et al., 2021; Roberts et al., 2021). Therefore, the discrepancies in the previous findings in this regard are somewhat expected. Iran experienced multiple peaks of the COVID-19 pandemic, leading to high mortality and the hospitalization of numerous patients and healthcare professionals. Therefore, the low level of resilience in the nurses of the present study could be due to their heavy workload, patient crowds, high mortality, and the smaller proportion of nurses to patients.

Two studies conducted with nurses in the Philippines indicated that nurses with higher resilience and who received more organizational and social support were at a lower risk of COVID-19 anxiety (Labrague and De los Santos, 2020; Labrague, 2021). Nursing researchers recommend implementing resilience training programs to enhance the psychological health of healthcare workers on an individual, professional, and organizational level (Chow et al., 2018). Resilient nurses will be able to resist stressors and feel capable of problem-solving in the stressful environment of hospitals (Mousavi, 2019). The stressful environment of the emergency department threatens the mental health of nurses, causes medication errors, reduces the quality of care, and even reduces the satisfaction and motivation of nurses. In addition to aggravating these mentioned problems, the COVID-19 pandemic caused nurses constantly worry about infecting themselves and their families with COVID-19 infection, which affected their concentration and accuracy (Alameddine et al., 2021). In this situation, nurses use a series of coping skills to adapt to this stressful situation, which does not necessarily lead to a favorable outcome. Resilience, or the capacity to “bounce back” or recover quickly after a stressful event, may help nurses manage, cope, and tolerate stressful situations (Labrague and De los Santos, 2020).

Our findings could raise the awareness of health authorities and managers regarding nurses’ resilience, fear, and anxiety so that effective interventions could be developed for increasing nurses’ resilience and reducing their fear and anxiety. One of the limitations of the present study was that some participants could not cooperate due to the crowdedness of the emergency room. The decrease in the severity of the Covid-19 pandemic has reduced nurses’ workload, so considering the mentioned limitations, we suggest that similar studies be conducted to evaluate nurses’ psychological distress and resilience.

## Conclusion

Based on the findings, the resilience score decreased significantly with the increase in fear and anxiety scores. Therefore, providing necessary training on dealing with psychological distress can increase resilience in nurses by reducing fear and anxiety.

## Data availability statement

The original contributions presented in this study are included in the article/supplementary material, further inquiries can be directed to the corresponding author.

## Ethics statement

The studies involving human participants were reviewed and approved by Kurdistan University of Medical Sciences. The patients/participants provided their written informed consent to participate in this study.

## Author contributions

NKK and RGG contributed in design and performing study. SD conducted data analysis. FD and SR contributed to grammar editing. All authors read and approved the final manuscript.

## Abbreviations

CDAS: Corona disease anxiety scale
CD-RISC: Connor-Davidson resilience scale
FCV-19S: fear of COVID-19 scale
WHO: World Health Organization.
